RETRACTED

# Design of Financial Risk Control Model Based on Deep Learning Neural Network

**DOI:** 10.1155/2022/5842039

**Published:** 2022-05-10

**Authors:** Donglai Yang, He Ma, Xiaoxin Chen, Lei Liu, Yuhang Lang

**Affiliations:** Saxo Fintech Business School, University of Sanya, Sanya 572000, Hainan, China

## Abstract

In recent years, with the continuous increase of financial business, the risk of business is on the rise. Among them, major risk cases are frequent, the cases are increasingly complex, and the means of committing crimes are concealed. The main research contents of this paper include the preprocessing of internal and external financial data and the structure design of recurrent NNs. Its purpose is to design a financial risk control model based on a deep learning NNs, thereby reducing financial risk. The Borderline-SMOTE algorithm is used first to preprocess the sample data, and the oversampling method is used to eliminate the imbalance of the data, and then, the long short-term memory deep NNs algorithm is introduced to process the sample data with time series characteristics. The final experiment shows that LSTM has a better accuracy, reaching 0.9715, compared with traditional methods; the sample preprocessing method and risk control model proposed in this paper have better ability to identify fraudulent customers, and the model itself has faster iteration efficiency.

## 1. Introduction

Risk control ability is mainly reflected in key nodes such as preloan approval, loan management, and postloan collection. As the first and most important risk control node in the financial process, preloan approval plays an obvious role. An excellent preloan approval capability can effectively help companies reduce the bad debt rate of financial services and can lower the lower limit of the qualifications of loan customers, thereby helping the rapid growth of financial business. Therefore, how to establish an effective prelending risk control model to reduce the risk of fraud by financial companies is a problem that every financial platform must solve, and it is also of great significance for promoting the sustainable development of the entire industry ecology.

At present, all walks of life are constantly developing and accumulating based on deep learning, forming their own industry-specific algorithms, thus solving many problems that could not be solved before. In the financial industry, deep learning methods have also been introduced to solve the problem of credit fraud. For credit fraud, it is necessary to prevent from the two dimensions of fraud and credit. In terms of fraud, malicious fraudulent loan behaviors must be identified, and in terms of credit, customers with poor qualifications and no repayment ability must be eliminated. In essence, this is still a process of identifying good customers and risky customers. If the occurrence of credit fraud cannot be prevented in time, it will often bring huge losses to the relevant financial institutions. In essence, this is still a process of identifying good customers and risky customers. If the occurrence of credit fraud cannot be prevented in time, it will often bring huge losses to the relevant financial institutions. In general, the benefits brought by a good customer are far less than the losses brought by a risky customer. From this point of view, a problem to be solved by financial risk control is actually a classification problem.

RETRACTED

The innovation of this paper is that (1) after in-depth understanding of the characteristics of various machine learning and deep neural networks, this paper builds a deep neural network model with better comprehensive performance based on long short-term memory neural network. (2) This model is different from the existing scorecard models that rely on statistical learning, which not only further reduces the dependence on financial experts but also has the ability to iterate rapidly. (3) After in-depth understanding of the characteristics of various machine learning (ML) and deep neural networks (NNs), this paper builds a deep NNs model with better comprehensive performance based on long short-term memory NNs. This model is different from the existing scorecard models that rely on statistical learning, which not only further reduces the dependence on financial experts but also has the ability to iterate rapidly.

## 2. Related Work

Remote control switches (RCS) can play an important role in reducing outage duration and cost. Izadi M's research shows that the model is treated as a multiobjective problem with two conflicting objectives, which is then solved by a nondominated sorting genetic algorithm II [1]. Although his research direction is forward-looking, it lacks reference value. The Judah G trial tested the impact on the adoption of two financial incentive programs based on principles of behavioral economics [2]. For the derivatives market, he proposed a new contingent claim for domestic or foreign derivatives markets. Jiang IM addresses the issue of hedging equity and exchange rate risk while making adjustments to protect the value of the collateralized equity [3, 4]. While his research provides a reference for companies' decisions when considering financing and investing in foreign markets, it lacks objectivity. Sarens G investigated the risk, risk management, and internal control information disclosed by companies in the country, by examining how and to what extent financial analysts in Belgium and Italy were scrutinized [5]. Dhar V proposed a new method to represent multiple simultaneous financial time series as images, motivated by deep learning methods for machine vision [6]. While this relationship helps bias learners toward learning what is useful to the application domain, it lacks comprehensiveness. The emerging availability of IoT devices, and the vast amount of data generated by such devices, could have a major impact on people's lives. Research by Morshed A shows that human progress in health medical diagnosis and prediction can be improved through the use of deep learning techniques [7].

RETRACTED

## 3. Financial Risk Control Model of Deep Learning NNs

### 3.1. System Architecture Design

All audit data come from the bank's big data platform (Hadoop). The analysis platform provides auditors at all levels with a visual operation tool to extract, clean, filter, filter, format, and analyze the massive data in the audit database. Using audit analysis, the powerful and flexible data analysis function of the platform enables further in-depth analysis of the data and finally forms the risk model of each business line. The model results will be displayed, processed, verified, counted, and summarized on the monitoring platform. The architecture of the intelligent risk control system is shown in Figure 1.

As shown in Figure 1, the intelligent risk control system obtains the data of various business systems of the bank from the big data platform, use the tools of the data analysis platform to analyze and process the extracted data, form the results of the risk model, and send the model results to the monitoring platform for dynamic risk monitoring and processing through the monitoring platform.

### 3.2. NNs Basics

#### 3.2.1. Overview of NNs

Neural networks are computational models inspired by biology. For biological neural networks, different neurons are connected to each other. The neural network in deep learning enables machines to imitate human activities such as audio-visual and thinking [8]. The scope of its role is shown in Figure 2.

The structure is shown in Figure 3.

On this basis, the back-propagation algorithm of the multilayer NNs is improved, that is, the BP NNs model [9, 10]. The back-propagation algorithm can improve the efficiency of adjusting parameters such as neuron weights, has strong learning ability, and is also one of the more popular NNs algorithms at present. Its model is shown in Figure 4.

#### 3.2.2. BP NNs Algorithm Flow

The entire NNs consist of the previous input layer (PIL), the middle HL (MHL), and the final output layer (FOL) [11]. The Sigmoid function is used in the introduction of the example, and its function and derivative forms are shown in formulas (1) and (2), respectively:

(1) $$\begin{array}{c} \text{f}\left(\text{x}\right)=\frac{1}{1+{\text{e}}^{-\text{x}}}, \end{array}$$

(2) $$\begin{array}{c} f^{\prime }\left(x\right)=f\left(x\right)\left[1-f\left(x\right)\right]. \end{array}$$

The algorithm is mainly divided into the following steps:

(1) Initialization parameters
Parameters such as weight thresholds are initialized by random numbers.
(2) Calculating the OL and HL neurons
According to the input feature *X*, the weight w1 of the IL and the HL, and the bias b1 between the IL and the HL, we obtain the intermediate value *Z* and the output *A* of the HL through the transformation function, and the corresponding formula is as follows (3):
  (3) $$\begin{array}{c} A_{j}=f\left(Z_{j}\right)\\ =f\left(\overset{n}{\underset{i=1}{\sum }}w1_{i,j}X_{i}+b1_{j}\right). \end{array}$$
(3) Calculating the output of the OL
According to the bias *b*2 of the HL and the OL, the weight w2 of the HL and the OL, and the input *A* of the HL, the result *y* of the OL is calculated, as shown in formula:
  (4) $$\begin{array}{c} y_{j}=\overset{n}{\underset{i=1}{\sum }}w2_{i,j}X_{i}+b2_{j}. \end{array}$$
(4) Calculation error
Calculate the mean square error according to the result *y* calculated in the forward propagation and the actual result Y in the data set, as shown in formula:
  (5) $$\begin{array}{c} e_{k}=\frac{1}{2}{\left(Y_{k}-y_{k}\right)}^{2}. \end{array}$$
(5) Modifying the weights and thresholds between neurons
Using the error er of each neuron in the OL and the output *y* of each neuron in the HL, the partial derivative operation is performed to update the weights *w*_1_ and *w*_2_, the thresholds are shown in following formulas:

(6) $$\begin{array}{c} \theta_{j}=\theta_{j}-\alpha J\left(\theta \right)\frac{\partial }{\partial \theta_{j}}, \end{array}$$

(7) $$\begin{array}{c} w1_{i,j}=w1_{i,j}+\alpha A_{j}\left(1-A_{j}\right)w_{j,k}\left(Y-y_{k}\right), \end{array}$$

(8) $$\begin{array}{c} w2_{i,j}=w2_{i,j}+\alpha A_{j}\left(Y-y_{k}\right). \end{array}$$

Similarly, the same chain derivation method is used to update the threshold b1 between the IL and the HL and the threshold b2 between the HL and the OL, as shown in following formulas:

(9) $$\begin{array}{c} b1_{j}=b1_{j}+\alpha A_{j}\left(1-A_{j}\right)V_{j,k}\left(Y-y_{k}\right), \end{array}$$

(10) $$\begin{array}{c} b2_{k}=b2_{k}+\alpha \left(Y-y_{k}\right). \end{array}$$

RETRACTED

### 3.3. Regularization Method

When the number of samples is too small or the model is too complex, overfitting will occur. In this case, the trained model can fit the training data well, but it performs poorly on the test set [12, 13]. Regularization methods prevent overfitting and improve model generalization performance by introducing additional information to the original model. Among them, the commonly used regularization methods are L1 regularization, L2 regularization, dropout regularization, etc. [14, 15].

#### 3.3.1. L1 Regularization (Lasso Regression)

L1 regularization actually adds the L1 regularization term to the original cost function, as shown in the following formula;

(11) $$\begin{array}{c} J=J_{0}+\frac{\lambda }{2b}{\left\|w\right\|}_{1}, \end{array}$$

where *J*_0_ is the original cost function in formula 11, *b* is the number of samples, *λ* is the regularization parameter, and *w* is the connection weight. Using the chain derivation method, the update function of the weight can be obtained as formula

(12) $$\begin{array}{c} \theta_{j}=\theta_{j}-\alpha \frac{\partial }{\partial \theta_{j}}J\left(\theta \right)-\frac{\alpha \lambda }{m}\mathrm{sgn}\left(\theta_{j}\right). \end{array}$$

The sgn function is a step function. When the weight is greater than 0, it returns 1, and when the weight is less than 0, it returns -1 [16, 17]. Generally speaking, in the process of L1 regularization being gradually strengthened, those feature parameters that carry less information and contribute little to the model will become 0 faster than the feature parameters that contribute more to the model, so L1 regularization is essentially a feature selection process [18]. The more L1 regularization is strengthened, the more feature parameters become 0, and the more sparse the parameters are, in order to prevent overfitting.

#### 3.3.2. L2 Regularization (Ridge Regression)

L2 regularization is similar in form to L1 regularization, as shown in the following formula:

(13) $$\begin{array}{c} \text{J}={\text{J}}_{0}+\frac{\lambda }{2\text{b}}{\left\|\text{w}\right\|}_{2}^{2}. \end{array}$$

Its weight update formula is shown in the following formula:

(14) $$\begin{array}{c} \theta_{j}=\left(1-\frac{\alpha \lambda }{m}\right)\theta_{j}-\alpha \frac{\partial }{\partial \theta_{j}}J\left(\theta \right). \end{array}$$

First calculate the square sum of each element of the vector and then take the square root according to the square sum to obtain the L2 norm. By minimizing the rule term |w| of the L2 norm, each element of *w* can be made small and close to 0. But unlike the L1 norm, it does not make the element equal to 0, but close to 0. It can also be seen from the L2 regularization formula that each iteration will make the weights keep getting smaller, thereby reducing the complexity of the model. Compared with L1 regularization, L2 regularization has the advantage of only reducing the proportion of weights to balance the weights without making the weights 0. This allows more features to play a role, and its stability is stronger than that of L1 regularization. The disadvantage is that it cannot obtain a sparse model like L1 regularization, and the sparse model will have better characteristics when dealing with high-dimensional samples.

RETRACTED

#### 3.3.3. RNN Training Process

RNN is divided into two training processes, forward propagation and back propagation, and iterates with timing as the core. The training process is as follows:

*(1) Forward Propagation*. Assuming that the input vector of the HL is *r*, the weight of the IL and the HL is *w*, the input vector is *x*, and the output vector of the HL at the previous moment is *q*, and then, the input vector of the HL at time *t* is as follows:

(15) $$\begin{array}{c} r_{n}^{t}=\overset{I}{\underset{i=1}{\sum }}w_{in}x_{i}^{t}+\overset{k}{\underset{k=1}{\sum }}w_{kn}q_{k}^{t-1}. \end{array}$$

The output vector of the HL at time *t* is as follows:

(16) $$\begin{array}{c} q_{n}^{t}=\theta_{\text{n}}\left(r_{n}^{t}\right), \end{array}$$

where *q* represents the output vector, and *θ* represents the HL activation function.

*(2) Back Propagation*. BPTT (back-propagation through time) is a commonly used algorithm for training RNNs. In essence, it is developed based on the BP algorithm. The training process is as follows:

Assuming that the error function is *E*, the error of the HL at time *t* can be obtained by chain derivation of the error *e* of node *j* as formula.

(17) $$\begin{array}{c} e_{n}^{\prime }=\theta^{\prime }\left(r_{n}^{t}\right)\left(\overset{k}{\underset{k=1}{\sum }}e_{k=1}^{k}w_{nk}+\overset{H}{\underset{n=1}{\sum }}e_{n=1}^{t+1}w_{nk}\right), \end{array}$$

where *e*_*n*_′ represents the error of the HL at time *t*, *e*_*k*_^*t*^ represents the error of the OL at time *t*, and *e*_*k*_^*t*+1^ represents the error of the HL at time *t*+1. Then, we take the derivation of the weight; here, we use the gradient descent method, and the derivation formula is as follows:

(18) $$\begin{array}{c} \Delta E\left({\text{w}}_{\text{i},\text{j}}\right)=\overset{\text{T}}{\underset{\text{i}=1}{\sum }}\text{e}w_{i}^{\prime }q_{i}^{\prime }. \end{array}$$

Then, according to the learning rate a, the weight adjustment formula is calculated as follows:

(19) $$\begin{array}{c} w_{i,j}=w_{i,j}^{\prime }+\Delta \alpha \left({\text{w}}_{\text{i},\text{j}}\right). \end{array}$$

RNN solves the problem of inability to memorize time series in BP NNs, but the network also has problems such as memory degradation, gradient explosion, or disappearance, which affect the prediction accuracy.

RETRACTED

## 4. LSTM Model Construction

### 4.1. LSTM Model Structure

This paper builds a model with one IL, three HL, and one OL. Next, taking the model with only one HL is an example to elaborate the algorithm flow of the LSTM model. Its model is shown in Figure 5.

Each LSTM layer contains a forget gate, an input gate (IG), and an output gate (OG). The goal of LSTM is to control the transmission of information through these three control gates to solve the gradient vanishing phenomenon that may occur in the NNs.

### 4.2. Parameter Adjustment and Optimization

We set the number of nodes in the input layer to 45, and the number of nodes in the output layer should be the same as the type of the output result. Regarding the setting of the number of hidden layers and the number of nodes, the determination method is relatively complicated. This paper adopts the method of choosing fewer layers or nodes at the beginning, and then gradually increases the complexity of the network structure, and takes the correct reflection of the relationship between the output and the input as the basic principle.

#### 4.2.1. Adjustment of the Number of Network Layers

For the four scenarios of one, two, three, and four hidden layers, the data in this paper are used to conduct experiments, and the loss curve on the test set is shown in Figure 6.

According to Figure 6, when the number of layers reaches 3, the LV becomes lower, while as the number of layers increases, the LV does not decrease significantly. The final loss, AUC, and KS values after model training are shown in Table 1.

It can be seen from Table 1 that the number of HL selected in this paper is 3. When the number of HL is 3, both AUC and KS reach high values.

#### 4.2.2. Activation Function Adjustment

Converting the input signal to the output signal is the main function of the activation function in the NNs structure. The NNs introduce nonlinear elements through the activation function and completes the nonlinear mapping. If the neuron does not go through the activation function, no matter how many HLs it goes through, the result of the final OL is a linear combination of the IL. Currently, commonly used activation functions are sigmoid, tanh, and ReLU. In this section, three activation functions are used to build the model, and the model effect of each activation function is verified.

In the experiment to confirm the effect of the activation function, other hyperparameters are also locked: the number of HLs is 3, and the number of nodes in each layer is (64, 32, 16). The activation function adopts sigmoid, tanh, and ReLU, respectively. For the above three models, the data in this paper are used to conduct experiments, and the loss curve on the test set is shown in Figure 7.

RETRACTED

According to Figure 7, when the activation function is sigmoid or tanh, the LV reaches a relatively low value, but the tanh function is not stable and there are many spikes. After all three models are trained, the final loss, AUC, and KS values are shown in Table 2.

It can be seen from Table 2 that the activation function selected in this paper is sigmoid, and both AUC and KS reach relatively high values when the activation function is sigmoid.

#### 4.2.3. Adjustment of Loss Function and Optimization Function

This paper uses two commonly used loss function: mean squared error function (mean squared error) and cross-entropy loss function (binary cross-entropy), and three commonly used optimization functions. During the experiment, other hyperparameters are still locked: the number of HLs is 3, the number of nodes in each layer is (64, 32, 16), and the activation function is sigmoid. Two loss functions and 3 optimization functions form a combination of 6 models. The loss curve on the test set is shown in Figure 8.

According to Figure 8, when the error function is MSE and the optimization function is Adam, the LV reaches a relatively low value. After all three models are trained, the final loss, AUC, and KS values are shown in Table 3.

It can be seen from Table 3 that the error function selected in this paper is MSE and the optimization function is Adam. When the error function is MSE and the optimization function is Adam, both AUC and KS reach relatively high values.

#### 4.2.4. Adjustment of Batch Size (Batch Size)

The so-called batch number refers to the number of data pieces used in each weight update of the model. At the same time, since the number of iterations required to run the complete data set decreases, the training speed will be further accelerated; however, if the batch size is too large, a local optimum may occur. If the batch size is too small, the randomness will become larger, and it is difficult to achieve the convergence effect, but it will have a better effect in individual cases. The loss curves under different batch numbers are shown in Figure 9.

In the experiment of confirming the effect of batch size, other hyperparameters are set as follows: the number of HLs is 3, the number of nodes in each layer is (64, 32, 16), and the activation function adopts sigmoid, respectively. The batch number is 50, 200, 1000, and 5000 in sequence. For the above four models, the data in this paper are used to conduct experiments, and the loss curve on the test set is shown in Figure 10.

RETRACTED

According to Figure 10, when the number of batches is 100, the loss value (LV) reaches a relatively low value, and when the number of iterations is about 17 times, the loss reaches a minimum value. After all four models are trained, the final loss, AUC, and KS values are shown in Table 4.

It can be seen from Table 4 that the batch number selected in this paper is 100 times. Different batch processing speeds have little effect on the AUC and KS values. A smaller batch number has better computing speed.

## 5. Financial Risk Experiment and Result Analysis

In this paper, the data set is divided by time span, which is commonly used in the financial field, and the data spanning half a year is divided into training set. Then, this data set is used for modeling. In this paper, all pseudorandom related parameters are fixed, and a 5-fold cross-validation method is used to reduce the randomness of the algorithm and make the detection results more stable. After all models are trained, the comparison results are shown in Table 5.

From the analysis in Table 5, it can be seen that as a simple classifier, logistic regression will be more popular than random forest, SVM, BP neural network, etc., at this stage, and the more effective classification algorithms proved in research are less effective. The XGBoost model, which is widely used in the field of risk control, and the LSTM model studied in this paper have better model effects than the above three models. We further analyzed the table and found that random forest has a better accuracy, reaching 0.9784. However, since the samples in our financial risk control field are all unbalanced samples, the accuracy rate can only be used as a reference and cannot represent the real performance of the model. Then, XGBoost has the highest F value, while the AUC and KS metrics of the LSTM model are higher. In comparison, the LSTM model is better than the XGBoost model currently used in the production environment. It may be because LSTM is more suitable for the unbalanced classification sequence problem of financial risk control, and can effectively process time series-related data. In order to further verify the effectiveness of LSTM as a classification model, the P-R graph and ROC graph are drawn as a reference, as shown in Figure 11.

Both ROC plots and P-R plots can be used to evaluate the generalization ability and classification ability of a model for a specific data set. It can be seen from the P-R diagram that in addition to the logistic regression model, other models perform well, and the random forest algorithm performs even better. However, it can be seen from the ROC diagram that LSTM has the largest area under the ROC curve, which can indicate that the LSTM model has a better classification effect. Moreover, when the random forest model and XGBoost model are not stable enough in practical applications, it takes a lot of time to adjust the parameters, and the cost of parameter adjustment is much greater than the LSTM model mentioned in this article. Therefore, the LSTM model in this paper has the best comprehensive effect and is suitable for use in the production environment.

RETRACTED

## 6. Conclusions

The structure of the original data of the People's Bank of China and the characteristic variables of financial risk control used in this paper. Then, the credit information data of the People's Bank of China are organized according to continuous variables and nominal variables, and are converted into numerical variables by one-hot coding according to the characteristics of the nominal variables. Finally, for the problem of missing values in the original data, in order to reduce the impact of a large number of missing values on the quality of the data set, this paper proposes to use the method of linear function normalization to preprocess the data, and fill in the features, and proposes the problem of data imbalance in the field of financial risk control. In this paper, all the data are divided into training set, validation set, and test set according to the time dimension segmentation method often used in financial scenarios. The analysis finds that the ratio of good customers to bad customers in the data set used is 21 : 1, and the data distribution is very unbalanced. In order to solve this problem, after processing the missing values, we use the Borderline-SMOTE algorithm to generate samplers, optimize the data imbalance problem, and use logistic regression, random forest, BP NNs, XGBoost, and other models to process the data. After in-depth understanding of the characteristics of various deep NNs, a financial risk control model based on LSTM is established. The LSTM model is a variant of RNN, which has a memory unit that can retain both short-term memory and some long-term memories. During training, the state of the IG, OG, and forgetting gate is changed to simulate the selective forgetting characteristics of human beings. The final effect of the LSTM model proposed in this paper has higher AUC and KS indicators than the traditional ML model XGBoost, and the actual cost of adjusting parameters is shorter, and the model update iteration is more convenient, suitable for use in production environments. The amount of data in the sample is very limited, and the consequence is that the analysis of some of the algorithms used in this article may not be accurate enough. In the future, it is necessary to continuously collect and accumulate new sample data to continuously verify and optimize the model generated in this paper.

RETRACTED

## Figures and Tables

**Figure 1:** Architecture of intelligent risk control system.

**Figure 2:** Deep learning application areas.

**Figure 3:** Artificial NNs element structure.

**Figure 4:** BP NNs structure diagram.

**Figure 5:** Single-layer LSTM model.

**Figure 6:** Loss curves under different layers. (a) Experimental results of one HL and two HLs. (b) Experimental results of three HLs and two HLs.

**Figure 7:** Loss curves under different activation functions.

**Figure 8:** Loss curves under different loss functions and optimization functions. (a) Cross-entropy loss function of two optimization functions. (b) Mean squared error function of two optimization functions.

**Figure 9:** Loss curves under different batch numbers. (a) Loss curve under batch number between 50 and 100. (b) Loss curve under batch number between 500 and 1000.

**Figure 10:** Loss curves under different batch sizes. (a) One HL and two HL loss curves. (b) Three HLs and four HL loss curves.

**Figure 11:** P-R and ROC diagrams. (a) P-R diagram. (b) ROC diagram.

**Table 1:** LOSS, AUC, and KS values under different layers.

Number of network layers	Training set			Test set		
	LOSS	AUC	KS	LOSS	AUC	KS
1	0.2696	0.8718	0.5826	0.3173	0.8260	0.5100
2	0.2086	0.9109	0.6695	0.2229	0.8501	0.5593
3	0.1 804	0.9297	0.7273	0.1925	0.8536	0.5578
4	0.1853	0.9361	0.7258	0.2295	0.8558	0.5553

**Table 2:** LOSS, AUC, and KS values under different activation functions.

Number of network layers	Training set			Test set		
	LOSS	AUC	KS	LOSS	AUC	KS
ReLU	0.3261	0.8442	0.5263	0.3225	0.7897	0.4696
Tanh	0.2594	0.8366	0.5397	0.2601	0.7916	0.4484
Sigmoid	0.0918	0.9669	0.8045	0.2101	0.7982	0.5664

**Table 3:** LOSS, AUC, and KS values under different error functions and optimization functions.

Loss function and optimized function composition	Training set			Test set		
	LOSS	AUC	KS	LOSS	AUC	KS
B_C-adam	0.0983	0.9646	0.7944	0.2179	0.8018	0.5844
B_C-sgd	0.6691	0.5659	0.1267	0.6654	0.5583	0.1329
B_C-RMSprop	0.1184	0.9499	0.7508	0.2295	0.7905	0.5692
MSE-a dam	0.0342	0.9585	0.7934	0.0580	0.8096	0.5863
MSE-sgd	0.2480	0.5990	0.1393	0.2473	0.5755	0.1452
MSE-RMSprop	0.0413	0.9425	0.7440	0.0444	0.7956	0.5760

**Table 4:** LOSS, AUC, and KS values under different error functions and optimization functions.

Number of batches (times)	Training set			Test set		
	LOSS	AUC	KS	LOSS	AUC	KS
50	0.0550	0.9976	0.9493	0.2272	0.8075	0.5555
100	0.0983	0.9646	0.7944	0.2179	0.801 8	0.5844
500	0.0705	0.9963	0.9307	0.2322	0.8118	0.5405
1000	0.0989	0.9946	0.9181	0.2300	0.7926	0.5054

RETRACTED

**Table 5:** Comparison of final results of different models.

Model	Acc	Precision	Recall	*F* value	AUC	KS
LR	0.7378	0.6909	0.7639	0.7256	0.7400	0.4801
RF	0.9784	0.9211	0.8295	0.8533	0.7887	0.6174
SVM	0.8853	0.8557	0.7981	0.8364.	0.7804	0.1080
XGBoost	0.9560	0.9127	0.8096	0.8937	0.7894	0.6189
BP	0.8298	0.6898	0.7597	0.8027	0.7397	0.5164
LSTM	0.9715	0.8609	0.8316	0.8712	0.8223	0.6363

## Data Availability

The data that support the findings of this study are available from the corresponding author upon reasonable request.
